This article has been retracted.

# p300 promotes proliferation, migration, and invasion via inducing epithelial-mesenchymal transition in non-small cell lung cancer cells

**DOI:** 10.1186/s12885-018-4559-3

**Published:** 2018-06-07

**Authors:** Xue Hou, Run Gong, Jianhua Zhan, Ting Zhou, Yuxiang Ma, Yuanyuan Zhao, Yaxiong Zhang, Gang Chen, Zhonghan Zhang, Shuxiang Ma, Xi Chen, Fangfang Gao, Shaodong Hong, Fan Luo, Wenfeng Fang, Yunpeng Yang, Yan Huang, Likun Chen, Haoxian Yang, Li Zhang

**Affiliations:** 1 Department of Medical Oncology, Sun Yat-sen University Cancer Center, 651 East Dongfeng Road, 510060 Guangzhou City, Guangdong Province People’s Republic of China; 2 State Key Laboratory of Oncology in South China, Guangzhou City, Guangdong Province People’s Republic of China; 3 Collaborative Innovation Center for Cancer Medicine, Guangzhou City, Guangdong Province People’s Republic of China; 4 Department of Medical Oncology, The Fifth Affiliated Hospital of Sun Yat-sen University, Zhuhai City, Guangdong People’s Republic of China; 5 Department of Clinical Research, Sun Yat-sen University Cancer Center, Guangzhou City, Guangdong Province People’s Republic of China; 6 Department of Thoracic Oncology, Sun Yat-sen University Cancer Center, 651 East Dongfeng Road, 637300 Guangzhou City, Guangdong People’s Republic of China

**Keywords:** Epithelial-mesenchymal transition, Invasion, Non-small cell lung cancer, p300, Prognosis

## Abstract

**Background:**

Histone acetyltransferase p300 is a crucial transcriptional coactivator and has been implicated as a poor prognostic factor in human cancers. However, little is known about the substantial functions and mechanisms of p300 in NSCLC proliferation and distant metastasis.

**Methods:**

We constructed p300 down-regulated and up-regulated cell lines through RNAi and recombinant plasmid transfection. Cell Counting Kit-8 assays were used to test the cell proliferation and confirmed by colony formation assays. Wound healing assays and transwell chamber assays were used to test the migration and invasion ability. Based upon these results, we measured the epithelial markers and mesenchymal markers after regulating p300 expression to explore epithelial-mesenchymal transition as a potential mechanism of p300 promoting NSCLC metastasis.

**Results:**

In NSCLC cells NCI-H1975 and NCI-H1993, down-regulation of p300 leads to inhibition of cell proliferation and colony formation. Cells with reduced p300 expression also demonstrate inhibited migration and invasion ability. Contrarily, up-regulation of p300 significantly enhanced the proliferation, colony formation, migration and invasion ability of NCI-H460. Importantly, further investigation shows that decreased p300 expression is associated with reduced expression of mesenchymal markers and increased expression of epithelial markers, while up-regulated p300 expression correlated with decreased expression of epithelial markers and increased expression of mesenchymal markers.

**Conclusions:**

As a crucial tumor promoter, p300 promotes cell proliferation, migration, and invasion in NSCLC cells. Epithelial-mesenchymal transition is a potential mechanism of p300 promoting NSCLC metastasis.

## Background

Non-small cell lung cancer (NSCLC) is the most prevalent malignancy and the leading cause of cancer death in the world, with a dismal 5-year survival rate of no more than 5% [1, 2]. Despite recent improvements in NSCLC diagnosis and therapy, most NSCLC patients die of invasion and metastasis to the regional lymph nodes and/or distant organs [3]. Unfortunately, the underlying mechanism for NSCLC invasion and metastasis remain poorly understood. Therefore, improved understanding of the molecular mechanisms underlying NSCLC invasion and metastasis is an urgent need for designing effective interventional strategies and prolonging patient life.

p300 is a member of the histone acetyltransferase family of transcriptional coactivators. It functions in the transcription process and catalyzes histone acetylation through its histone acetyltransferase activity [4–6]. Furthermore, p300 can also acetylize some transcriptional factors, such as p53 [7], HIF-1α [8], c-Myb [9], and STAT-1 [10], thus participating in epigenetic regulations of some genes involved in DNA repair, cell growth, differentiation, and apoptosis. Investigations in breast cancer, colorectal cancer, and gastric cancer have identified p300 as a tumor suppressor [11, 12]. However, several studies suggest that p300 promotes cancer progression and that its expression correlates with the tumorigenesis of several human cancers [13–15]. Over-expression of p300 is a poor prognostic factor in breast cancer, prostate cancer, hepatocellular carcinoma, and esophageal squamous cell carcinoma [15–18]. Our previous study investigated the value of p300 expression in surgically resected NSCLC patients, and we found that low p300 expression was an independent prognostic marker of better survival in operable NSCLC patients [19]. However, the functions and mechanisms of p300 in NSCLC proliferation and metastasis need to be investigated comprehensively.

In this present study, we explored the functions of p300 in NSCLC proliferation, invasion, and metastasis through regulating the p300 expression in vitro. We further investigated the gene expressions of epithelial markers and mesenchymal markers after regulating p300 expression, to explore epithelial-mesenchymal transition as a potential mechanism of p300 promoting NSCLC metastasis.

## Methods

### Cell culture and regents

This study was approved by the Ethics Committee of Sun Yat-sen University Cancer Center. The human NSCLC cell lines NCI-H292 (ATCC CRL-1848), NCI-H460 (ATCC HTB-177), PC-9 (RRID:CVCL_B260), A549 (ATCC CCL-185), NCI-H1650 (ATCC CRL-5883), NCI-H1993 (ATCC CRL-5909), NCI-H1975 (ATCC CRL-5908), HCC827 (ATCC CRL-2868), and NCI-H1299 (ATCC CRL-5803) were obtained from the State Key Laboratory (SKL) of Oncology in South China. These cells grew at 37 °C in a humidified atmosphere of 95% air and 5% CO2 using Dulbecco’s modified Eagle’s medium supplemented with 10% fetal bovine serum.

### Western blot analysis

Western blot analysis of protein expression was performed as described previously [20]. Briefly, protein lysates (20 μg) were separated using sodium dodecyl sulfate-polyacrylamide gel electrophoresis, and target proteins were detected using Western blotting with antibodies against p300 (1:500, Abcam); E-cadherin (1:1000, CST); Vimentin (1:1000, CST); Snail (1:500, CST); Fibronectin (1:100,Merck Millipore); β-catenin (1:1000, CST); and GAPDH (1:1000, CST).

### Construction of p300 down-regulated cells

HEK-293 T cells were seeded in 6 well plates and grown to 40–60% confluence. According to the manufacturer’s instructions, Lenti-sip300 (shp300) and negative control (shNC) with package vectors were transfected into HEK-293 T cells for 72 h. The sequences of the p300 shRNA, which were designed and synthesized by the Sigma-Aldrich Company (Shanghai, China), were as follows: sense, 5’-CCGGGCCTTCACAATTCCGAGACATCTCGAGATGTCTCGGAATTGTGAAGGCTTTTTG-3′, and antisense, 3’-GGCCCGGAAGTGTTAAGGCTCTGTAGAGCTCTACAGAGCCTTAACACTTCCGAAAAAC-5′. The shNC were used as the control group, and the sequences were as followed: sense, 5’-CCGGGC TTCTCCGAACGTGTCACGTCTCGAGATGTCTCGGAATTGTGAAGGCTTTTTG-3′, and antisense, 3’-GGCCCGAAGAGGCTTGCACAGTGCAGAGCTCTACAGAGCCTTAACACTTCCGAAAAAC-5′.

Lentivirus supernatants were harvested and used to infect NCI-H1975 cells or NCI-H1993 cells with 2 μg/ml polybrene for 48 h. The cells were cultured with 2 μg/ml puromycin in the medium for a week, and constructed p300 down-regulated cells H1975/shP300 and H1993/shP300, as well as negative control cells H1975/shNC and H1993/shNC.

### Construction of p300 up-regulated cells

NCI-H460 cells were seeded in 6 well plates and grown to 80% confluence before plasmid transfection. P300-pcDNA3.1-EGFP (P300) or scrambled plasmid (Vector) was transfected using Lipofectamine 2000 (Invitrogen) as per the manufacturer’s instructions. The Lipofectamine- DNA compound was added to cell medium for 6 h and then changed to normal medium. After 48 h, we constructed p300 up-regulated cells H460/P300 and control cells H460/Vector, the expression of P300 was assessed by western blotting.

### Cell proliferation assay

Cell proliferation was measured by a Cell Counting Kit-8 (Dojindo, Kumamoto, Japan). Cells were plated in 96-well plates at a density of 2 × 10^4^ cells/mL, maintained at 37 °C in a humidified atmosphere of 95% air and 5% CO2. Twenty-four hours later, 10 ul of CCK-8 solution was added to each well. After incubation for 1 h, the absorbance was determined at 450 nm using a microplate reader.

### Colony formation assay

Colony formation assay was performed as described previously [20]. Briefly, 48 h after shRNA transfection, cells were trypsinized, resuspended as single cells, and plated in 6-well plates with 500 cells per well. After 7–10 days of culture, the colonies were fixed with methanol and stained with 1% crystal violet for 10 min. Colonies with more than 50 cells were counted under the microscope.

### Cell invasion assay and wound healing assay

Invasion assays were performed with Transwell system (Corning® BioCoat™ Matrigel® Invasion Chambers with 8.0 μm PET Membrane in two 24-well plates). Briefly, 5 × 10^4^ cells were resuspended in serum-free medium and added to the upper inserts. 750 μl medium supplemented with 10% FBS was added in the lower chamber as a chemoattractant. After incubation for 24–72 h, cells migrating to the bottoms of the filters were stained with a three-step stain set (Thermo Fisher Scientific), and the number of cells was counted under the microscope. Cell migration was also assessed with wound healing assay. Confluent cells were scraped by 200 μl pipette tip to create an artificial wound, and incubated in fresh medium containing Mitomycin C (5 μg/ml) for 12 h. Migration distance was measured by taking pictures at 0 and 12 h.

### Statistical analysis

Mean values of paired data were compared with the Student t-test. Analysis of variance was used to examine two groups’ data with continuous variables. Categorical data were analyzed with either the Fisher exact or χ2 test. Each experiment was conducted independently at least three times, and values were presented as the means ± standard error of the mean (SEM) unless otherwise stated. The statistical analyses were performed using the SPSS software program (version 21.0; IBM Corporation). Statistical significance was indicated by a conventional *p* value less than 0.05.

## Results

### Differential expressions of p300 in NSCLC cells

We first measured the p300 expression level in nine NSCLC cell lines: NCI-H292, NCI-H460, PC9, A549, NCI-H1650, NCI-H1993, NCI-H1975, HCC827, and NCI-H1299. Western blot analysis demonstrated that p300 expression was higher in NCI-H1975 and NCI-H1993, and lower in HCC827 and NCI-H460 (Fig. 1a). To investigate the role of p300 in NSCLC cells, we constructed down- and up-regulated NSCLC cells. We used lenti-sip300 (shp300) with package vectors to generate p300 down-regulated NSCLC cells H1975/shP300 and H1993/shP300, while negative control (shNC) with package vectors to generate control cells H1975/shNC and H1993/shNC (Fig. 1b). We used P300-pcDNA3.1-EGFP to transfect NCI-H460 cells to generate p300 up-regulated cells H460/P300, while scrambled plasmid to generate control cells H460/Vector (Fig. 1c).

**Fig. 1:** **a** Relative p300 expression of nine aggressive non-small cell lung cancer cell lines were examined with Western Blot analysis; **b** NCI-H1975 and NCI-H1993 cells were transfected with shp300 and shNC, western blot was used to determine interference efficiency; **c** P300-pcDNA3.1-EGFP and scrambled plasmid were transfected into NCI-H460, western blot was used to determine transfection efficiency

### Regulation of p300 affected the proliferation and colony formation of NSCLC cells

We performed a CCK-8 Assay to assess the effect of p300 on NSCLC cell viability. Proliferation was reduced in H1975/shP300 compared with H1975/shNC at 48 and 72 h (*p* < 0.0001, both; Fig. 2a). The same result was observed in H1993/shP300 and H1993/shNC (*p* < 0.001 at 48 h, *p* < 0.0001 at 72 h; Fig. 2b). Conversely, proliferation was increased in H460/p300 compared with H460/Vector at 12 and 24 h (*p* < 0.0001, both; Fig. 2c). To evaluate a longer-term impact, we performed colony formation assays on H1975/shP300, H1993/shP300, and H460/P300 cells as well as control cells. As expected, down-regulation of p300 significantly decreased the clonogenic ability of both cells, clone numbers were 263 ± 37, and 363 ± 16 for H1975/shP300 and H1975/shNC (*p* < 0.01), 218 ± 20 and 341 ± 19 for H1993/shP300 and H1993/shNC, respectively (*p* < 0.01) (Fig. 2d). Contrarily, up-regulation of p300 increased colony formation of H460, with clone numbers of 196 ± 6 for H460/P300 and 56 ± 7 for H460/Vector (*p* < 0.001) (Fig. 2e).

**Fig. 2:** Effects of p300 regulation on the proliferation and colony formation of NSCLC cells. **a** Cell proliferation measured by a Cell Counting Kit-8 Assay were significantly reduced in H1975/shP300 compared with H1975/shNC at 48 and 72 h, *p* < 0.0001; **b** Cell proliferation were significantly reduced in H1993/shP300 compared with H1993/shNC at 48 h (*p* < 0.001) and 72 h (*p* < 0.0001); **c** Cell proliferation were significantly increased in H460/P300 compared with H460/Vector at 12 and 24 h, *p* < 0.0001; **d** Colony formation assays showed clone numbers were significantly reduced in H1975/shP300 and H1993/shP300 compared with H1975/shNC and H1993/shNC (*p* < 0.01); **e** Clone numbers were significantly increased in H460/P300 compared with H460/Vector (*p* < 0.001)

### Regulation of p300 affected the migration and invasion of NSCLC cells

We evaluated the effects of p300 on cell migration and invasion of NSCLC cells. We first examined the cell migration using wound healing assay. H1975/shP300 demonstrated slower motility (wound closure) compared with H1975/shNC (*p* < 0.01, Fig. 3a), while H460/P300 demonstrated increased motility compared with H460/Vector (*p* < 0.001, Fig. 3b). Furthermore, we investigated whether regulation of p300 expression would inhibit NSCLC cell invasion. Transwell chamber assays showed that transient transfection of p300 shRNA dramatically reduced the invasion of H1975 and H1993 cells compared with normal control cells, invasive cell numbers on the membrane were 111 ± 26 and 253 ± 24 for H1975/shP300 and H1975/shNC (*p* < 0.001), 217 ± 35 and 369 ± 9 for H1993/shP300 and H1993/shNC, respectively (*p* < 0.001) (Fig. 3c). Contrarily, up-regulation of p300 increased the invasion of H460, with invasive cell numbers on the membrane of 1028 ± 92 for H460/P300 and 426 ± 33 for H460/Vector (*p* < 0.01, Fig. 3d).

**Fig. 3:** Effects of p300 regulation on the migration and invasion ability of NSCLC cells. **a** Wound healing assay demonstrated that migration distance of H1975/shP300 were smaller than H1975/shNC (*p* < 0.01); **b** Wound healing assay demonstrated that migration distance of H460/P300 were larger than H460/Vector (*p* < 0.001); **c** Transwell chamber assays demonstrated that invasive cell numbers on the membrane were significantly reduced in H1975/shP300 and H1993/shP300 compared with H1975/shNC and H1993/shNC (*p* < 0.001); **d** Transwell chamber assays demonstrated that invasive cell numbers on the membrane were significantly increased in H460/P300 compared with H460/Vector (*p* < 0.01)

### p300 expression was positively correlated with epithelial-mesenchymal transition (EMT)

In order to explore the mechanism of p300 expression increasing migration and invasion abilities of NSCLC cell lines, we measured the levels of EMT-related markers. Compared with normal control cells, increased expression of epithelial markers E-cadherin, and reduced expression of mesenchymal markers Vimentin, and Snail were demonstrated in H1975/shP300 cells (Fig. 4a), while reduced expression of E-cadherin and increased expression of Fibronectin and β-catenin were demonstrated in H460/P300 (Fig. 4b). These results suggested p300 expression correlated positively with EMT and thus promoted cell migration and invasion.

**Fig. 4:** Effects of p300 regulation on the epithelial and mesenchymal markers expression of NSCLC cells. **a** Changes of epithelial and mesenchymal markers expression of H1975/shP300 compared with H1975/shNC; **b** Changes of epithelial and mesenchymal markers expression of H460/P300 compared with H460/Vector

## Discussion

Histone acetyltransferase p300 was found to play an important role in DNA repair, cell growth, differentiation, and apoptosis through epigenetically regulating some transcriptional factors; thus much research in recent years has focused on its function in malignant tumorgenesis and progression [11–18]. We previously explored p300 expression in resected NSCLC tissues and correlated it with patients’ clinicopathological features as well as survivals. We found that low expression of p300 was an independent prognostic factor of better disease-free survival and overall survival in operable NSCLC patients [19]. That result was consistent with findings in other human malignancies, such as esophageal squamous carcinoma [16], prostate cancer [18], and hepatocellular cancer [17], indicating p300 playing an important role in tumor progression, although some other studies demonstrated p300 as a tumor suppressor in breast cancer [12] and gastric cancer [11]. Based on the above findings, we designed the current research to comprehensively investigate the functions of p300 in NSCLC cell lines.

In this study, we investigated the function of p300 in NSCLC proliferation, invasion, and metastasis. After down-regulating the p300 expression in vitro through transfecting p300 shRNA into NSCLC cell lines, we found reduced proliferation in a CCK-8 assay, and significantly decreased clonogenic ability in colony formation assay. Furthermore, down-regulation of p300 dramatically inhibited cell migration in wound healing assay and cell invasion in Transwell chamber assay. Collectively, knockdown of p300 in NSCLC cell lines led to inhibition of cell proliferation, migration, and invasion. Contrarily, up-regulating the p300 expression in vitro through transfecting P300-pcDNA3.1-EGFP significantly enhanced the proliferation, migration and invasion ability of H460. Mechanically, reduced p300 expression correlated with increased expression of epithelial markers and decreased expression of mesenchymal markers, while up-regulated p300 expression correlated with decreased expression of epithelial markers and increased expression of mesenchymal markers, suggesting EMT as a potential mechanism of p300 promoting cell migration and invasion. However, the limitation of our study is that we have not confirmed the conclusion in in vivo experiment, and we will plan it in our future work.

Our findings on p300 function in NSCLC cell lines confirm the results of our previous study in resected NSCLC tissues [19]. Down-regulated p300 leads to inhibited NSCLC proliferation, migration, and invasion capacity in vitro, indicating its role as a promoter in NSCLC progression. Consistently, patients with higher expression of p300 in tumor tissue are at higher risk of distant metastasis and shorter survival after complete resection, which is independent of conventional TNM staging system. Integrating our serial findings in vitro and in patients’ clinical outcomes, the function of p300 has been elucidated in promoting NSCLC invasion and metastasis.

The mechanism of p300 promoting cancer progression is attributed to its role as a transcriptional coactivator in previous study [7–10]. p300 acetylates histones, weakens their interaction with the DNA, loosens the nucleosome, and facilitates different transcription factors access to the DNA template [21]. By interacting with androgen receptor (AR) and activating AR-dependent transcription, p300 promotes AR-dependent prostate cancer progression, which can be blocked by siRNA against p300 [18, 22]. p300 also mediates androgen-independent transactivation of the AR by IL-6 in AR-independent prostate cancer [23]. MYC is another proto-oncogene whose transcription is activated by p300, and targeting p300 could repress MYC transcription and thus inhibit cancer cell progression [24]. Above all, p300 acts as a transcriptional coactivator of many oncogenes and plays an important role in human cancers. In our current study, we find interestingly that EMT might be another mechanism of p300 promoting NSCLC invasion and metastasis. After down-regulating p300 expression in NCI-H1975, expressions of epithelial markers E-cadherin, β-catenin were increased, and expressions of mesenchymal markers Vimentinand Snail were decreased, while up-regulating p300 expression in NCI-H460 correlated with reduced expression of E-cadherin and increased expression of Fibronectin and β-catenin. These changes represent key molecular features of EMT, which was regarded as initial events in the process of tumor metastasis. This result demonstrated that knockdown of p300 led to loss of mesenchymal phenotype, and acquisition of epithelial phenotype, while up-regulated of p300 led to acquisition of mesenchymal phenotype and loss of epithelial phenotype. This observation explains the results of function research in vitro, and also consistent with our previous study in human NSCLC tissues, which found that patients with high expression of p300 were under higher risk of distant metastasis after complete resection. Since p300 induces EMT, cancers with higher p300 have more potential to detach from primary tumor and metastasis to distant organ.

Mechanisms of p300 inducing EMT have been studied in other groups. Snail is thought to be a substrate whose histones in promoter could be acetylated by p300 and expression be up-regulated, and thus leads to reduced expression of E-cadherin [25]. ZEB1 is demonstrated to bind p300 and promotes the formation of p300-Smad transcriptional complex, then activity of ZEB1 is enhanced, synthesis of E-cadherin is reduced, and finally EMT occurred [26]. Since the current studies of p300 regulating EMT focus on the transcriptional level, we think it is also necessary to explore the mechanisms comprehensively on post-transcriptional protein regulation, which would be the direction of our future work.

## Conclusions

In this current study, we demonstrate that p300 plays an important role in proliferation, migration, and invasion of NSCLC cells. We further find epithelial-mesenchymal transition as a novel mechanism underlying the invasive properties of NSCLC cells with high p300 expression. Therefore, targeting p300, or histone acetyltransferases inhibitors, might be a potential therapeutic strategy for blocking NSCLC metastasis.

## Abbreviations

AR: androgen receptor
CCK-8: Cell Counting Kit-8
EMT: epithelial-mesenchymal transition
HAT: histone acetyltransferases
NSCLC: non-small cell lung cancer
shRNA: small hairpin RNA
siRNA: small interfering RNA
